# Profound Effect of Pulmonary Surfactant on the Treatment of Preterm Infants with Respiratory Distress Syndrome

**DOI:** 10.1155/2022/4166994

**Published:** 2022-10-03

**Authors:** Lin Liu, Quanmin Deng

**Affiliations:** Department of Pediatrics, People's Hospital of Deyang City, Sichuan, Deyang 618000, China

## Abstract

Inherited diseases caused by dysfunction of pulmonary surfactant metabolism or surfactant dysfunction have recently been considered the underlying causes of neonatal and pediatric respiratory diseases. Respiratory distress syndrome in premature infants is a common respiratory disease in pediatrics. It is caused by underdeveloped lungs in infants and a lack of active substances on the surface of the alveoli, which leads to insufficiency of lung function, which can lead to difficulty breathing, increased heart rate, facial bruising, and more. Neonatal Respiratory Distress Syndrome is a very dangerous disease with a high mortality rate and a great threat to children's lives and health. Therefore, enough attention and treatment should be caused in clinical practice. Natural pulmonary surfactant (PS) has achieved positive effects in the treatment of neonatal respiratory distress syndrome (RDS), reducing neonatal mortality, the application of mechanical ventilation, and the occurrence of late complications. To further explore the role of pulmonary surfactants in the treatment of neonatal respiratory distress syndrome, to analyze the best time to use PS to prevent RDS, this paper has selected premature infants with RDS received by the neonatal department of a hospital in a province from March 2019 to October 2020 to compare the efficacy of pulmonary surfactant (PS) in preterm infants with respiratory distress syndrome (RDS). The experiment has found that the average mechanical ventilation time (5.1 d) and oxygen therapy time (7.3 d) in the early group are shorter than the average mechanical ventilation time (6.4 d) and oxygen therapy time (10.6 d) in the late group. It has been demonstrated that early administration of pulmonary surfactant (PS) therapy is of great help in improving respiratory distress syndrome in premature infants.

## 1. Introduction

Perinatal medicine is a kind of work that starts from the period when the pregnant woman is diagnosed as pregnant and carries out a series of works such as protection and nursing accessories, as well as examination for the pregnant woman. With the continuous improvement of perinatal medical technology, increasingly premature infants survive, but premature infants are a high-risk group for intraventricular hemorrhage (IVH). Some external factors such as inappropriate mechanical ventilation, bad stimulation, incorrect endotracheal suction, asphyxia, and infection are all incentives for the occurrence of IVH. Pulmonary surfactant refers to a complex lipoprotein secreted by alveolar type II epithelial cells, which is distributed on the surface of the alveolar liquid molecular layer between the liquid and air interfaces. For preterm infants, especially within 32 weeks, the survival rate is significantly higher than other preterm infants; NRDS is a common disease. The reason for this is progressive dyspnea caused by the lack of pulmonary surfactant (PS), resulting in decreased alveolar surface tension and alveolar collapse. For a long time, PS replacement therapy has become the best method for the treatment of NRDS, but in the process of clinical use, it is found that the treatment strategies for PS vary greatly due to the difference of neonatal gestational age. The purpose of this article is to retrospectively analyze the cases of RDS prevention in premature infants with respiratory distress syndrome, and to explore the necessity of using PS in children.

Preterm birth serves as a major cause of newborn infant morbidity and mortality. Because maternal age at birth provides the most significant factor for predicting unfavorable newborn consequences, there is a great deal of interest in strategies to delay preterm birth. Studies on hemostatic drugs have shown that COX inhibitors (e.g., indomethacin) are more effective than other drugs in delaying labor, but findings on the outcomes of neonates exposed to these drugs before birth have been controversial. Indomethacin has also been used postpartum for the drug treatment of patent ductus arteriosus (PDA), but there are no data on the effect of prenatal exposure on postpartum ductal patency. While Doni D primarily focused on the relationship between prenatal indomethacin (AI) and postnatal ductus arteriosus patency, it has been concluded that PDA is more common at low gestational age, thus reducing the incidence of PDA could improve overall outcomes in preterm neonates [1]. Inhaled nitric oxide (iNO) therapy is useful for the treatment of managed respiratory stress and acute episodes of hypoxemia. Yet, these advantages have not been confirmed in infants born precociously (<34 weeks). The aim of Alvarado Socarras et al. were to present the experience of eight precocious infants with respiratory distress syndrome (RDS) and intractable hypoxemia, all of whom had a history of oliguria. These newborns were treated with iNO to prevent their death. As a result, all fetuses were found to have improved oxygenation. Neonates showed evidence of high-flow lung and were verified by ultrasound echocardiography. Five babies born prematurely survived without treatment-related comorbidities. Two died of hemorrhage in the lungs secondary to the ductus arteriosus, and the other died of pneumonia. Thus, iNO therapy is available for a subsection of high-risk episodes of prematurity due to hypoxemia, but not widely used [2]. Pan et al. investigated the clinical efficacy of intratracheal infusion of pulmonary surfactant (PS) combined with budesonide in the prevention of bronchopulmonary dysplasia (BPD) in very low birth weight (VLBW) infants. He randomly assigned 30 VLBW infants less than 32 weeks gestational age with neonatal respiratory distress syndrome (NRDS) (grades III–IV) due to intrauterine infection with PS plus budesonide or PS alone. It was found that endotracheal infusion of PS coupled with budesonide was effective in reducing the occurrence of BPD in VLBW preterm infants with severe NRDS [3]. Dietrich et al. compared the impact of two different surfactant delivery schedules on cerebral oxygenation in preterm infants: LISA (low invasive surfactant delivery method) and InSurE (intubation SURfactant delivery, and extubation). Serial studies were performed on consecutive subjects by near infrared spectroscopy (NIRS), measuring regional cerebral oxygen saturation (rSO_2_C) and calculating partial cerebral oxygen extraction efficiency (cFTOE). NIRS data were recorded 30 minutes before surfactant administration (T0), during surgery (Tproc), and at 30 minutes (T1), 60 minutes (T2), and 120 minutes (T3) after surgery. It was found that SpO_2_ decreased substantially at Tproc compared to T0, T1, T2, and T3. rSO2C decreased temporarily with the LISA and InSurE procedures, and the decrease was greater in the LISA group. Consistently, cFTOE increased simultaneously in the LISA group, higher than in the insured group, suggesting that it represented a reparative mechanism [4].

Acute respiratory distress syndrome is a medical condition with a very high death rate in the world today, and many scholars have studied this area. Nin et al. analyzed the association between hypercapnia present within 48 hours of initiation of mechanical ventilation and outcomes in patients with acute respiratory distress syndrome (ARDS). A secondary study of 3 prospective nondisruptive Cochrane research studies focused on 927 patients with ARDS in intensive care units (ICUs) in 40 countries. The association with maximum PaCO_2_ and mortality within the first 48 hours showed that mortality was higher when PaCO_2_ was ≥50 mmHg or higher. Severely hypercapnic patients (PaCO_2_ ≥ 50 mmHg) had a higher rate of complications, more organ collapse, and a worse prognosis. It is concluded that severe hypercapnia seems to be indirectly linked to better ICU mortality in patients with ARDS [5]. Fierro et al. have evaluated the development of an extracorporeal membrane oxygenation (ECMO) program for the treatment of adults with acute respiratory distress syndrome (ARDS). A descriptive study was performed on 15 cases treated between 2010 and 2016 since the program was approved [6]. Data on mechanical ventilation (MV) characteristics and radiological characteristics of H7N9-induced ARDS cases are still lacking. Hui and Zhi described the MV and radiographic characteristics of adult patients with microbiologically confirmed ARDS caused by H7N9 admitted to the ICU within 3 months. All patients presented with ventilatory failure with acute respiratory distress syndrome (ARDS) and required MV in the intensive care unit. Four patients received intensive care due to incurable hypoxemia and required extra resuscitative treatment. Despite these measures, three patients died. It was concluded that low tidal volume tactics were the norm in ARDS patients with H7N9 infection [7]. In the related work section, these studies analyzed in detail the incidence of respiratory distress syndrome in preterm infants. There is no denying that these studies have greatly promoted the development of related fields. However, there are relatively few studies on the in-depth role of pulmonary surfactants in the treatment of premature infants with respiratory distress syndrome, and it is necessary to fully explore these aspects in the research in this field.

This paper has mainly explored the in-depth impact of pulmonary surfactants on the treatment of preterm infants with respiratory distress syndrome. In the comparison of the mortality rate of children in the early group and the late group, it was found that, within 28 days after birth, 2 patients died in the early group (the 3rd and 4th days after birth), and 1 patient died in the late group (the 3rd day after birth), both of them died of pulmonary hemorrhage. Early or late administration of pulmonary surfactant (PS) did not significantly affect mortality. In contrast, the mean periods of organic oxygenation (5.1 d) and oxygen therapy (7.3 d) were shorter in the early stage group than in the late stage group (6.4 d) and oxygen therapy (10.6 d). It has been shown that the early administration of pulmonary surfactant (PS) treatment can significantly improve the duration of mechanical ventilation and oxygen therapy in premature infants. However, in the early group and the late group, the incidence of complications such as NEC, PDA, air leakage, pulmonary hemorrhage, and severe IVH was between 2 and 7, and there was no significant impact. The pulmonary function indexes PaO_2_, PaCO_2,_ a/A, PO_2_, OI, and PH in the early and late groups after treatment were significantly better than those in the control group.

## 2. Methods for the Treatment of Premature Infants with Respiratory Distress Syndrome

Respiratory distress syndrome (NRDS) in premature infants is caused by a lack of surfactant and tissue hypoplasia in the lungs. The natural course of the disease begins within two days of birth, and if not treated in time, it can lead to death due to hypoxia and respiratory failure, which is the cause of death in about 50–70% of premature infants [8]. As shown in Figure 1, from the data of European neonatal NRDS, it can be seen that NRDS has many complications and high mortality, posing a great threat to its survival [9].

The development of the lung consists of five stages: embryonic, glandular, tubular, vesicular, and alveolar stages [10]. Early neonatal lung development is still in the vesicle stage and has not yet developed. Insufficient or no secretion of PS can cause insufficient expansion of alveoli, impair pulmonary ventilation and respiratory function, and develop RDS. Because RDS can cause serious complications, once diagnosed, active treatment is required. Intratracheal instillation of PS is the first choice for the treatment of premature infants with RDS [11]. In addition, it is necessary to take measures such as mechanically assisted ventilation and inhalation of hyperoxia, and these measures are likely to cause adverse events such as barotrauma, oxygen toxicity, and infection in children. Tissue fibrosis develops and develops into bronchopulmonary dysplasia (BPD) in premature infants [12].

Respiratory failure refers to severe impairment of lung ventilation and/or air exchange due to various causes. The inability to maintain adequate air exchange at rest causes (or does not result in) hypoxemia, resulting in a series of pathophysiological changes and corresponding clinical symptoms [13]. Diagnosis of respiratory failure is usually confirmed by blood gas analysis: at sea level, at rest, and breathing, when the patient's arterial partial pressure of oxygen (PaO_2_) is less than 60 mmHg, and the partial pressure of carbon dioxide does not exceed 50 mmHg, respiratory failure can be diagnosed, but to rule out causes such as anatomical cardiac drainage and reduced cardiac output. It is divided into acute and chronic phases. Acute respiratory failure is a very dangerous respiratory disease with a mortality rate of over 60% [14]. The details are shown in Table1.

The pulmonary respiratory membrane is composed of 6 layers including the liquid molecular layer containing alveolar surfactant, the alveolar epithelium, the epithelial cell basement membrane, the space between the capillaries and the alveoli, the capillary basement membrane, and the capillary endothelium. The normal lung respiratory membrane regulates the fluid in the lungs, ensuring dryness of the alveoli and adequate filling of the interstitium. The stability of the lung respiratory membrane determines the absorption of oxygen and the normal excretion of carbon dioxide. When the inflammatory response is not controlled, it leads to the destruction of the alveoli, capillary epithelium, endothelial cells, and basement membrane, resulting in abnormal interstitial filling [15]. Fluid infiltration and poor perfusion result in pulmonary interstitial edema, which is a massive infiltration of alveoli by fluid, protein, and blood cells, as well as decreased alveolar surfactant, alveolar collapse, increased respiratory membrane thickness, and decreased alveolar surface area. This results in breathing problems, hypoxia, decreased lung compliance, and increased pulmonary blood pressure [16].

In computer image preprocessing, image enhancement is a very effective method. The traditional image intensification methods primarily include the spatial domain method and transform domain method, as shown in Figure 2 [17]. The spatial domain method mainly performs direct operation processing on the pixel gray value in the spatial domain, such as image grayscale transformation, histogram correction, image spatial domain smoothing and sharpening, and pseudo-color processing. The transform domain method refers to processing the transformed values of the image in a specific transform region. An indirect method is used, where the Fourier transform is first performed, then the frequency domain is filtered, and finally the filtered image is inversely transformed back into the spatial domain to obtain an enhanced image.

Medical X-ray image enhancement is an important subject in the field of image processing and the basis of image processing. The purpose of image enhancement is to emphasize the relevant information in the image, weaken or delete the unnecessary content, to strengthen the useful information and facilitate the identification and interpretation [18].

X-ray imaging system is a comprehensive system composed of optics, microelectronics, precision machinery, image acquisition and processing, computer, and other disciplines [19]. It is shown in Figure 3.

The SSR algorithm is a single-scale Retinex method, which has the advantages of simplicity, easy implementation, no need for scene correction, significantly faster operation speed, and clear physical meaning [20].

The mathematical form of the SSR algorithm is as follows:

(1) $$\begin{array}{c} O_{i}\left(x,y\right)=\log I_{i}\left(x,y\right)-\log\left[F\left(x,y\right)*I_{i}\left(x,y\right)\right]\text{.} \end{array}$$

Among them, *O*_*i*_(*x*, *y*) is the output of Retinex in the ith color spectrum. *I*_*i*_(*x*, *y*) is the image distribution, that is, the luminance value at the location of (*x*, *y*). *∗* represents the convolution operation. *F*(*x*, *y*) is a wraparound function, as follows [21]:

(2) $$\begin{array}{c} F\left(x,y\right)=CF^{\prime }\left(x,y\right)\text{.} \end{array}$$

Among them, *F*′(*x*, *y*) is the basic form of the surrounding function, and C is the normalization factor, that is, it satisfies:

(3) $$\begin{array}{c} \iint F\left(x,y\right)dxdy=1\text{.} \end{array}$$

C can be calculated by the formula:

(4) $$\begin{array}{c} C=\frac{1}{\sum \sum F^{\prime }\left(x,y\right)}\text{.} \end{array}$$

According to the Retinex theory, it represents the spatial distribution of the illuminance image and the distribution of the scene reflection image, then:

(5) $$\begin{array}{c} I_{i}\left(x,y\right)=L_{i}\left(x,y\right)e_{i}\left(x,y\right)\text{.} \end{array}$$

The logarithm of both sides of the formula is taken and the terms are shifted to get:

(6) $$\begin{array}{c} \log\;\left(e_{i}\left(x,y\right)\right)=\log\;\left(I_{i}\left(x,y\right)\right)-\log\left(L_{i}\left(x,y\right)\right)\text{.} \end{array}$$

The convolution term in the SSR algorithm can be regarded as a calculation method of spatial illumination. Its physical meaning is to eliminate the effect of illumination changes by calculating the ratio of the pixel to the weighted average of its surrounding area. The mathematical form of formula (1) ensures that the color is constant, and its form can be as follows:

(7) $$\begin{array}{c} O_{i}\left(x,y\right)=\log\frac{l_{i}\left(x,y\right)e_{i}\left(x,y\right)}{\bar{l_{i}\left(x,y\right)}\bar{e_{i}\left(x,y\right)}}\text{.} \end{array}$$

The convolution term is expressed as the product of the illuminance and the spatially weighted mean of the reflection, so if,

(8) $$\begin{array}{c} l_{i}\left(x,y\right)\approx l_{i}\left(x,y\right). \end{array}$$

That is, the spatial variation of illuminance is relatively gentle, then:

(9) $$\begin{array}{c} O_{i}\left(x,y\right)\approx \log\frac{e_{i}\left(x,y\right)}{\bar{e_{i}\left(x,y\right)}}\text{.} \end{array}$$

It can be seen that in the approximate case, the output of Retinex does not depend on the influence of illumination.

### 2.1. The Form of the Environmental Function

Inverse square surround form:

(10) $$\begin{array}{c} F^{\prime }\left(x,y\right)=\frac{1}{r^{2}}\text{,}\\ r=\sqrt{x^{2}+y^{2}.} \end{array}$$

It is in turn modified to depend on space constants of the form:

(11) $$\begin{array}{c} F^{\prime }\left(x,y\right)=\frac{1}{1+r^{2}/k_{1}^{2}}\text{.} \end{array}$$

The wraparound function in Gaussian form is as follows:

(12) $$\begin{array}{c} F^{\prime }\left(x,y\right)=e^{-r^{2}/k_{2}^{2}}\text{.} \end{array}$$

Various environmental functions are used to conduct experiments on a large number of chest radiographs. The results show that the Gaussian type has a good dynamic range compression ability. Among them, the Gaussian surround function has the most significant enhancement effect on image details.

### 2.2. Subsequent Processing of Output Results

The results obtained from formula (1) have both positive and negative conditions, so to obtain suitable printing and display effects, subsequent processing is also required.

Through the analysis of multiple chest images, a histogram that approximates the normal distribution is obtained, which conforms to the normal distribution of the natural image histogram. If straight line stretching is used, the obtained image will be shallow, and the improvement effect of the chest image will be poor. However, after truncating both ends of the histogram, the effect of image processing can be significantly improved, as shown in Figure 4.

The interception and stretching of the output result can be expressed by formula (13), where *I*_*i*_ and *I*_*o*_ are the input and output, respectively. *x*_*m*_ represents the dynamic range of the output device, such as 255 for an 8 bit system (that is 2^8^ − 1), and *I*_*hi*_ and *I*_*low*_ are the upper and lower intercept points, respectively.

(13) $$\begin{array}{c} I_{o}=\left\{\begin{array}{c} 0I_{i}\leq I_{low}\\ \frac{I_{i}-I_{low}}{I_{hi}-I_{low}}x_{m}\\ x_{m}I_{i}\geq I_{hi} \end{array}\right)I_{low}<I_{i}<I_{hi}\text{.} \end{array}$$

The selection of the upper limit intercept point *I*_*hi*_ and the lower limit intercept point *I*_*low*_ is the key.

X-ray medical images were processed using different methods. Sometimes, the captured photos will have strong contrast, making people feel unnatural. An offset based on the average of the original image can be added to the grayscale.

## 3. Experimental Design of the Deep Effect of PS on the Treatment of Preterm Infants with Respiratory Distress Syndrome

### 3.1. Source and Nature of Cases

For the convenience of research, this paper selected 90 premature infants with NRDS who were hospitalized in the Neonatal Intensive Care Unit (NICU) of a Provincial Hospital from March 2019 to October 2020. The details are shown in Table 2.

The diagnostic criteria of NRDS are progressive dyspnea and central cyanosis within 6–12 hours after birth. Chest X-ray showed specific manifestations such as ground-glass changes, air bronchus sign, or white lung, and clinical or imaging evidence confirmed RDS grade III or IV. The parents of the investigated children all agreed to use pulmonary surfactant replacement therapy.

### 3.2. Exclusion Criteria

Exclusion criteria: congenital hereditary metabolic disorder, fatal congenital heart disease, critically ill children with massive pulmonary hemorrhage, intracranial hemorrhage, shock when hospitalized; premature infants more than 8 hours before hospitalization; death during treatment or a family member's petition to wait for treatment.

### 3.3. Etiological

The pathogenesis of NRDS is that the alveolar type II epithelial cells are not fully developed, the production and release of surfactants are reduced, and normal respiratory needs cannot be met, resulting in a clinical syndrome of a series of symptoms. The main components of PS are dipalmitoyl lecithin and surface-active binding protein. The former accounts for more than 60%, and the latter accounts for about 10%. PS on the molecular surface of the alveolar liquid phase causes the alveoli to show a decrease in tension and stabilizes the lung blasts, to keep the liquid in the alveolar capsules from leaking into the alveoli.

### 3.4. Treatment Options

#### 3.4.1. General Treatment

The three groups of children were given tracheal intubation and mechanical ventilation immediately after the clinical manifestations or diagnosis was confirmed. Ventilation parameters were individually adjusted according to the patient's condition. Routine symptomatic and supportive treatment was performed concurrently with mechanical ventilation. It mainly includes: ensuring that the children in each group are kept away from noise pollution, giving the children a warm box adjusted to the appropriate temperature and humidity to keep the children warm, maintaining the body temperature within the normal range, using the same type of antibiotics to prevent infection (if necessary), paying attention to the children's water, electrolyte, acid-base, fluid balance, paying attention to circulatory function, and closely monitoring vital signs such as breathing, heart rate, blood pressure, and transcutaneous oxygen saturation. To ensure good perfusion of each tissue, if necessary, drugs were used for positive inotropy, improving vascular function and microcirculation perfusion for children. The children were given nutritional support treatment, and parenteral nutrition was active in the early stage. Generally, the initial intravenous fluid volume of children was 70–80 ml/kg/d. The amount of fluid replacement is adjusted according to body weight, blood sodium, etc., to avoid large fluctuations in body weight.

For the amount of amino acids, 2∼2.5 g/kg/d can be supplemented on the first day of illness to maintain nitrogen balance, supply enough glucose, amino acids, fat emulsion, trace elements, etc., and supply enough calories as soon as possible. Gradually enteral feeding was started at the same time. When necessary, blood gas analysis should be performed to understand the child's physical condition and regular head color. Doppler ultrasound and fundus screening should be performed to assist in diagnosis and treatment; and bleeding should be prevented.

### 3.5. Notes

It takes a period of time for PS to be completely absorbed after being inhaled into the lungs, so the child should take a supine position within 6 hours after injection and should not turn over, or suck sputum. Unless there is obvious airway obstruction, it should be delayed for 12–24 hours. For 6 hours after administration, it should be turned every 3 to 4 hours. For children with edema, the body position should be appropriately changed to promote pulmonary circulation and relieve orthostatic edema.

The clinical manifestations of the patients were closely monitored: (1) Monitoring of SPO, T, P, R, BP, blood gas analysis, and chest X-ray examination. (2) Be gentle when doing various operations to reduce adverse stimulation to the child, such as too loud sound, too much light, and too frequent postures. The intravenous fluid is kept at a constant rate, and the rectal temperature is kept at 36.5∼37.0°C to avoid excessive body temperature changes, which will lead to cardiovascular dysfunction, thereby affecting the effect of PS.

When using drugs, some children will develop bruising, slow heart rate, and decreased blood oxygen saturation. They need to immediately use a resuscitation bag to pressurize oxygen or use a ventilator for mechanical ventilation. In addition, adjusting the posture during drug use can make the drug distribution in the lungs more even, so that the neck will be involved, which will cause the excitation of the vagus nerve, which will cause the heart rate to slow down and the heart to stop beating.

### 3.6. Indications for Weaning

The patient's condition was basically stable, with spontaneous breathing ability and regular rhythm, FiO_2_ < 30%, PEEP decreased to 3–4 cm H_2_O, and arterial blood gas was basically normal: PaO_2_ > 50 mmHg, PaCO_2_ < 45 mmHg. Acid-base balance: when PH is 7.25∼7.35, nCPAP and endotracheal intubation can be removed and mechanically assisted ventilation therapy can be removed. It is noted that dexamethasone should be statically pushed to reduce laryngeal edema before weaning from mechanical ventilation. If necessary, intravenous gamma globulin can be given to enhance immunity to prevent infection.

## 4. Data Analysis of PS in the Treatment of Preterm Infants with Respiratory Distress Syndrome

Comparison of the overall conditions of the three groups: the control group adopted the methods of sputum suction, oxygen inhalation, keeping warm, improving pulmonary microcirculation, mechanical ventilation, preventing complications, and protecting liver and kidney functions. The PS treatment group was given early (1.50.4) hours, and the PS treatment group was given late (6.02.3) hours. The details are as follows: in the supine position, the right lateral position, the left lateral position, and the supine position, the drug solution is instilled into the lower trachea. After 1 body position, the balloon was compressed and breathed for 1∼2 m in 40∼60 times/min. The severity of maternal hormone use, birth weight, and RDS did not differ significantly (*P* > 0.05) among the three groups, as shown in Table 3. The general maternal, pregnancy, and prenatal conditions are presented in Table 4.

Figure 5 is a comparison of the mortality of children in the early group and the late group.

As can be seen from Figure 5, within 28 days after birth, 2 people in the early group (birth days 3 and 4) died due to pulmonary hemorrhage. In the late group, 1 died from pulmonary hemorrhage (3 days after birth); 1 in the early group died 28 days after birth due to sepsis, and 2 in the late group died from NEC.

Figure 6 shows the duration of ventilatory ventilation and oxygen therapy for children in the early and late groups. It can be seen from Figure 6 that the mean length of mechanical ventilation (5.1 d) and oxygen therapy (7.3 d) was shorter in the early group than in the late group (6.4 d) and oxygen therapy (10.6 d) after excluding the early death cases.

The incidence of complications in the early group and late group is shown in Figure 7.

As can be seen from Figure 7, the number of cases of NEC, PDA, air leakage, pulmonary hemorrhage, severe IVH, and other complications in the early group and the late group was not much different. Therefore, it can be concluded that the early application of PS can significantly reduce the ventilator ventilation time and oxygen therapy time in premature infants with RDS. However, there was no significant effect on complications and mortality in preterm infants with RDS.

The lung function comparison of the three groups is shown in Figure 8. Among them, the evaluation of pulmonary function indicators include: alveolar partial pressure of oxygen (PaO_2_), arterial partial pressure of carbon dioxide (PaCO_2_), and oxygenation index (OI). The clinical efficacy comparison of the three groups of children is shown in Table 5.

It can be seen from Figure 8 that the lung function indexes of the early group and the late group were greatly improved after treatment. The results have shown that pulmonary surfactant has an obvious clinical effect on neonatal respiratory distress syndrome, which can significantly improve the pulmonary function of children and shorten the treatment time.

## 5. Conclusion

NRDS is the most common respiratory disease in neonates, which has a serious impact on the healthy growth and life safety of neonates. This paper has found through analysis that NRDS is mainly seen in premature infants and children born to diabetic mothers. The lower the gestational age, the higher the prevalence. Due to the lack of PS, the alveoli are compressed, resulting in atelectasis, resulting in a short circuit of blood gas in the lung, which reduces PaO_2_ and oxygenation. Clinically, progressive dyspnea occurs, and the fatality rate is still high. Early respiratory intervention for children is the key to the treatment of respiratory distress syndrome and can improve the prognosis of children. Due to pulmonary hypoplasia, the lungs do not open, the pulmonary fluid transport is blocked, and pulmonary edema, cell damage, progressive respiratory failure, etc., easily lead to a variety of complications. It is an important factor leading to neonatal death. In the experiment, it was found that the morning and evening of PS treatment did not affect the incidence of related complications. However, PS replacement therapy strategies and dosing methods are also constantly improving. In addition to therapeutic administration, there is also prophylactic administration. Postpartum prophylactic administration of PS to preterm infants with a high risk of RDS within 30 minutes after delivery can significantly reduce the incidence and severity of RDS, and significantly reduce neonatal mortality and air leakage.

## Figures and Tables

**Figure 1:** European neonatal statistics.

**Figure 2:** Classification of image augmentation methods.

**Figure 3:** X-ray imaging system.

**Figure 4:** Schematic diagram of intercepted stretching.

**Figure 5:** Comparison of the mortality rate of children in the early group and the late group.

**Figure 6:** Comparison of mechanical ventilation time and oxygen therapy time between two groups of children in the early group and late group.

**Figure 7:** Complications in children.

**Figure 8:** Pulmonary function of the three groups of children.

**Table 1:** Diagnostic criteria for acute respiratory distress syndrome.

Diagnostic parameters		Diagnostic criteria
Mode of onset		Known clinical impairment, new or worsening respiratory symptoms within 1 week of acute onset
Chest imaging		Decreased translucency of both lungs—cannot be made by pleural effusion, lobar opacification/pulmonary atelectasis, or nodules completely
Causes of pulmonary edema		Explained
Oxygenation	Mild	Oxygenation index: 200∼300, and PEEP/CPAP ≥ 5 cm H_2_O
	Moderate	Oxygenation index: 100∼200, and PEEP/CPAP ≥ 5 cm H_2_O
	Severe	Oxygenation index: ≤100, and PEEP/CPAP ≥ 5 cm H_2_O

**Table 2:** Basic information of respondents.

Parameters	Number of cases	
	90	
	Male	Female
	43	47
Gestational age	29.5–34 2 w	30.0–35.2 w
Body weight	0.90–2.20 kg	1.20–2.3 kg

**Table 3:** Comparing the overall condition of children in the three groups.

		Control group (*n* = 30)	Early group (*n* = 30)	Late stage group (*n* = 30)
Hormone use before birth (cases)		20	24	22

Birth weight (cases)	<1000 g	3	3	3
	1001∼1600 g	18	17	18
	1601∼2300 g	9	10	9

RDS (cases)	Level III	20	19	26
	Level IV	10	11	14

**Table 4:** Comparison of general conditions of mothers during pregnancy and prenatal period among the three groups.

Pregnancy and obstetric conditions	Control group	Early group	Late stage group
Gestational hypertension (number of cases)	3	3	3
Gestational diabetes mellitus (number of cases)	2	3	3
Chorioamnionitis (number of cases)	0	1	0
Antenatal infection (number of cases)	7	6	6
Intrauterine distress (number of cases)	2	2	1

**Table 5:** Comparison of clinical efficacy of three groups of children.

Group	Healing	Significantly effective	Effective	Invalid
Control group (number of cases)	6	9	6	8
Early stage group (number of cases)	17	8	4	1
Late group (number of cases)	17	7	4	2

## Data Availability

No datasets were analyzed during the current study.
